# SERR-U-Net: Squeeze-and-Excitation Residual and Recurrent Block-Based U-Net for Automatic Vessel Segmentation in Retinal Image

**DOI:** 10.1155/2021/5976097

**Published:** 2021-08-09

**Authors:** Jinke Wang, Xiang Li, Peiqing Lv, Changfa Shi

**Affiliations:** ^1^Rongcheng College, Harbin University of Science and Technology, Rongcheng 264300, China; ^2^School of Automation, Harbin University of Science and Technology, Harbin 150080, China; ^3^Mobile E-Business Collaborative Innovation Center of Hunan Province, Hunan University of Technology and Business, Changsha 410205, China

## Abstract

**Methods:**

A new SERR-U-Net framework for retinal vessel segmentation is proposed, which leverages technologies including Squeeze-and-Excitation (SE), residual module, and recurrent block. First, the convolution layers of encoder and decoder are modified on the basis of U-Net, and the recurrent block is used to increase the network depth. Second, the residual module is utilized to alleviate the vanishing gradient problem. Finally, to derive more specific vascular features, we employed the SE structure to introduce attention mechanism into the U-shaped network. In addition, enhanced super-resolution generative adversarial networks (ESRGANs) are also deployed to remove the noise of retinal image.

**Results:**

The effectiveness of this method was tested on two public datasets, DRIVE and STARE. In the experiment of DRIVE dataset, the accuracy and AUC (area under the curve) of our method were 0.9552 and 0.9784, respectively, and for SATRE dataset, 0.9796 and 0.9859 were achieved, respectively, which proved a high accuracy and promising prospect on clinical assistance.

**Conclusion:**

An improved U-Net network combining SE, ResNet, and recurrent technologies is developed for automatic vessel segmentation from retinal image. This new model enables an improvement on the accuracy compared to learning-based methods, and its robustness in circumvent challenging cases such as small blood vessels and intersection of vessels is also well demonstrated and validated.

## 1. Introduction

The essence of automatic segmentation of retinal vessel image is to classify the vessel pixel and its surrounding pixels. In clinical application, manual segmentation of retinal vessel is time-consuming and labor-intensive, which is also highly dependent on clinician's experience. With the explosion of retinal image data, computer-aided segmentation of retinal vessels has attracted more and more attention [1]. Currently, automatic retinal vessel segmentation methods can be divided into two categories: machine learning- (ML-) based and deep learning- (DL-) based approaches.

For the unsupervised ML-based method, Chaudhuri et al. [2] designed a 2D Gaussian matched filter for the retinal vascular segmentation, and then, other methods based on vascular morphology and specific rules of pixels emerged, such as the morphological processing method proposed by Yang et al. [3], which first enhanced vascular features and suppressed background information, and then utilized fuzzy clustering to achieve vascular segmentation. Zhao et al. [4] proposed a deformable model-based method, which used the regional information of different vascular types to fulfill segmentation. Li et al. [5] optimized the matched filtering method for vascular segmentation and width estimation. In summary, the unsupervised ML-based method is known for fast speed, but it tends to result in low precision.

For the supervised ML-based methods, thanks to the manually labeling process, the training model is much strengthened, and thus, it is more reliable than unsupervised ML methods in vascular feature extraction. Staal et al. [6] used the KNN algorithm to classify each pixel, compared the features in the training set with the corresponding feature in the test set, and extracted the most similar top *k* data, so as to obtain the classification with the highest frequency. Soares et al. [7] first used a 2D filter to extract the overall features of the retinal image and then employed the naive Bayes to classify the retinal background and vessels. Ricci and Perfetti [8] extracted the green channel of retinal image in preprocessing and then employed SVM for segmentation according to the difference of vascular width. Fraz et al. [9] proposed a method of combining AdaBoost and Bagging algorithms, which integrates the feature vectors with the binary classification model, and using the supervision method to perform automatic analysis of retinal images. In general, the accuracy of supervised ML-based method is greatly improved; however, it cannot properly adapt to the shape, scale, and geometric transformation of blood vessels and thus tend to result in low robustness in the segmentation of small vessels and their intersections.

For the DL-based methods, due to the improvement of computer hardware, these approaches are able to provide accurate prediction of vascular and nonvascular pixels, with the description of vascular scale, shape, and multiple curvature information. Among them, the Convolution Neural Network- (CNN-) based method has been attracted extensive attention by scholars, and thanks to its ability of automatically extracting feature information from high-dimensional dataset. Fu et al. [10] used Fully Convolutional Networks (FCN) to produce a vessel probability map and obtained high accuracy and sensitivity on the DRIVE and STARE datasets. Mo and Zhang [11] used an auxiliary classifier in the middle layer of CNN to solve the vanishing gradient problem. Jiang et al. [12] proposed a modified end-to-end deep FCN to improve the accuracy of small blood vessel segmentation. Dharmawan et al. [13] provided a new blood vessel data enhancement method and combined it with U-Net to improve the accuracy of segmentation.

With the development of semantic segmentation [14], many DL-based network models have been proposed. These models confirm that deeper networks are more suitable for image segmentation tasks [15]. However, problem such as the vanishing gradient makes it difficult to train deep models. One solution is to utilize the optimized activation function (e.g., ReLU or ELU) for such problem [16]. Another method is proposed by He et al. [17], who used the function mapping to train a deep residual model to overcome this problem.

## 2. Related Work

We briefly review the related works, including U-Net, recurrent block, ResNet, and Squeeze-and-Excitation.

### 2.1. U-Net

Among numerous methods of medical image segmentation, U-Net [18] is considered to be one of the most successful methods, which is composed of convolutional encoder and decoder unit, with several advantages for segmentation tasks. First, it allows the use of both global features and context information. Second, it can accomplish the training work with limited samples and achieve prior performance. Third, it processes the entire image end-to-end and generates the segmentation result directly. The above three characteristics ensure U-Net retains the complete context information of the input image, which is a great advantage compared with other patch-based methods [19].

### 2.2. Recurrent Block and ResNet

Different improved models of U-Net model have also been proposed. Compared with traditional U-Net, the performance of the network training has been improved, with superior convergence. Meanwhile, the promotion of skip connection for medical image segmentation task has also been verified. Specifically, by adding recurrent structure [20], the network level of U-Net is deepened, and a superior learning effect is acquired by stacking several ordinary convolution blocks. In addition, to solve the network optimization problem, the residual network (ResNet) is proposed [21], which makes it possible to train CNN more deeply. Lian et al. [22] proposed a globally and locally enhanced residual U-Net for accurate retinal vessel segmentation, and the experimental results of the network on two datasets proved the effectiveness of the method.

### 2.3. Squeeze-and-Excitation

Squeeze-and-Excitation net is a new network structure proposed by Hu et al. [23]. It automatically acquires the importance of each feature channel via learning, captures features according to this importance, and discards features that are not important to the current task. Although the structure increases the number of parameters and calculation burden in the original classification network, it achieves better results. Based on the fusion of fully connected and multiplicative features, SE could implement an attention mechanism. Guo et al. [24] proposed a residual spatial attention network (RSAN) for the retinal vessel segmentation, which not only be used to construct a deep network for deriving more complex vessel features, but also effectively eliminates overfitting problem.

The proposal of abovementioned semantic-level networks provides new ideas for the segmentation of retinal vessels and become important theoretical basis of the proposed method. This paper leverages the above technologies to propose a new end-to-end automatic segmentation framework for retinal vessels.

The main contributions of this paper are as follows:

- On the basis of the U-Net network, the convolutional layers of the upsampling and downsampling parts are modified, and the recurrent block is used to increase the network depth and obtain higher segmentation accuracy
- The residual module is used to alleviate the vanishing gradient problem caused by the increased network depth, promote the model to converge faster, and achieve the purpose of training a deeper network
- By introducing attention mechanism into the U-shaped network, SE structure can adaptively extract the retinal image features, while suppressing irrelevant regions, ensuring that the network can focus on features related to the blood vessel segmentation task

The rest of the paper is organized as follows: Section 3 introduces the image preprocessing and the proposed network architecture; Section 4 focuses on the experimental results and analysis; Section 5 discusses and summarizes the whole paper.

## 3. Method

In this paper, we propose a SERR-U-Net for retinal vessel segmentation, which consists of two main steps: (1) image preprocessing and (2) proposed network architecture.

### 3.1. Image Preprocessing

For the best learning efficiency and higher accuracy, the image is preprocessed first, with the flowchart shown in Figure 1.

#### 3.1.1. Detail Enhancement

The retinal images used are RGB images. In order to improve the accuracy of segmentation, this paper uses the ESRGAN method [25] to preprocess the retinal images, which is a popular perceptual-driven method for single-image super-resolution reconstruction. By this means, the contrast of the retinal image increases, the gap between the contour of the vessel and the background is sharpened, and the noise is reduced, which is beneficial to the subsequent vascular segmentation. Furthermore, the Contrast Limited Adaptive Histogram Equalization (CLAHE) algorithm is employed to enhance local contrast.

#### 3.1.2. Grayscale Conversion

The original color retinal image was separated into 3 channels: red (R), green (G), and blue (B).  Figure 2 provides some examples. It can be seen that among all the channel results, the green channel shows less noise and high contrast between the vessel and the background; therefore, the green channel is selected as the input data.

#### 3.1.3. Image Intensity Transformation

For the green channel of the retinal image, first, standardized processing is adopted to perform data centralization, thereby increasing the generalization ability of the model. Then, the normalization process is used to make the data distributed between 0 and 1, so as to realize the unification of the measurement. Finally, nonlinear gamma transformation is used to adjust the illumination intensity of the input retinal images and perform a nonlinear operation on the intensity values, which makes the intensity values of the input and output image constitute an exponential relationship:

(1) $$\begin{array}{c} V_{\text{out}}=AV_{\text{in}}^{\gamma }, \end{array}$$

where *A* is a constant, and in the common case of *A* = 1, the input and output values are typically in the range [0, 1]. *V*_in_ represents the grayscale value of the input image and takes a value in the range [0, 1]. *γ* denotes the grayscale scaling factor, which is used to stretch the image grayscale. Through nonlinear gamma transformation, the overexposed or too dark retinal images are corrected.

#### 3.1.4. Data Augmentation

Due to the relatively small amount of training data, data augmentation is performed to reduce the influence of overfitting. In this paper, the retinal images are rotated at random angle to simulate different acquisition environments, and moreover, patches are extracted from 20 DRIVE and 10 STARE training images via random cropping. As a result, a set of 285,000 patches is generated.  Figure 3 shows an example of random cropping results of retinal images.

### 3.2. Proposed Network Architecture

The proposed SERR-U-Net (our code is available at https://github.com/lixiang007666/SERR-U-Net-Retinal-Vessel-Segmentation) in this paper is a modification of U-Net. It is inspired by SE, ResNet, and traditional recurrent network and refers to some ideas from the recurrent residual CNN-based U-Net (R2U-Net) [26]. The Conv+ReLU structures of the U-Net encoder and decoder are changed to SE-ResNet module and recurrent block structure. Since the network depth is increased, the residual structure of ResNet is used to avoid the vanishing gradient problem caused by the increased network depth.

Figure 4 provides the framework of the proposed SERR-U-Net. Firstly, the codec of U-Net is replaced with the Conv+ReLU structures, and meanwhile, the SE-ResNet module and recurrent blocks are added, which inherits the symmetrical characteristic of the U-Net. Similarity, the hidden layer is also composed of a downsampling part and an upsampling part. The difference is that, when skipping and connecting, instead of U-Net cropping and splicing, a cascading operation based on feature summation of different time steps is adopted to obtain more features of lower level.

The detailed parameters of the SERR-U-Net are listed in Table 1. The network includes two parts: encoder and decoder, each of which consists of multiple blocks. The encoder block contains three parts: a convolution layer, an SE block, and a maximum pooling layer. Each convolution layer is followed by a BN and a ReLU processing. The structure of the decoder block is similar to the encoder block, except that it employed a transposed convolutional layer instead of the pooling layer. Based on the above framework, the parameter number we used is 370,817 in all.

This paper proposes a combination structure of the SE-ResNet module and the recurrent module. First, a recurrent module is added to the common “Conv+ReLU” layer, and then, the structure is stacked. Through this processing, a deeper network is obtained, which is conducive to higher accuracy. Second, a residual structure was inserted between the input layer and the output layer, which could avoid the vanishing gradient problem effectively as the network depth increases. Lastly, based on the above structure, we modify the traditional ResNet module to SE-ResNet module, so as to introduce attention mechanism. This structure can properly fit the complex correlation between channels and reduce the number of parameters and calculation burden caused by the increased network depth.

Figure 5 shows the two most important parts of attention mechanism: full connection layer and feature multiplication fusion. Suppose that the input image *H* × *W* × *C* is stretched into dimension of 1 × 1 × *C* through global pooling and full connection layer and then multiplied by the original image, and meanwhile, each channel is given the corresponding weight to achieve the purpose of feature fusion. In addition, in the denoising task, each noise point is assigned a weight, the low-weight noise points are automatically removed, while the high-weight noise points are retained, and the parameter calculation is reduced. This is why the SE module is considered as an attention mechanism.

The proposed network allows the use of global positioning to obtain context information at the same time, which is appropriate for retinal image segmentation. The pipeline architecture at each level allows the global information of the model to be retained. Besides, the added recurrent module could effectively increase the depth of the network, while the SE residual module solves the vanishing gradient problem, and the added attention mechanism reduces the difficulty of understanding the model during training.

Considering that in the practical process of retinal images, the image dataset may be blurred or deformed due to factors such as illumination, weather, and the shaking of the collection equipment, which results in difficult follow-up processing. In order to optimize low-quality pictures, the ESRGAN [25] technology was utilized in this paper to generate realistic textures in super-resolution processing of single image and meanwhile suppress artifacts.

### 3.3. Loss Function

The purpose of the segmentation of the retinal vascular images is to classify the pixels as vessels and background in the images. However, since almost 90 percent pixels of the retinal image belong to the background, while the other 10 percent belong to the vessels [27], thus the training of the network is likely to stop at a local optimal value, and the segmentation target would be more inclined to the background. In view of such imbalance problem, *Dice* coefficient [19] is more suitable than CE (Cross-Entropy); therefore, *Dice* coefficient was chosen as the loss function for the network optimization, which we aim to minimise. A differentiable approximation of *Dice* loss is defined as follows:

(2) $$\begin{array}{c} L_{\text{dice}}=1-\frac{2\sum_{i}^{N}\;p_{i}g_{i}}{\sum_{i}^{N}\;p_{i}^{2}+\sum_{i}^{N}\;g_{i}^{2}}, \end{array}$$

where *p*_*i*_ represents a vector of the predicted binary segmentation and *g*_*i*_ represents a vector of the ground truth. By employing the above loss function, the complicated process of defining weight coefficients could be avoided.

Moreover, in order to eliminate the instability of the loss values and the validation dataset during the training process, BN (Batch Normalization) layer and L2 regularization are added into the framework in this paper to avoid the occurrence of overfitting. The purpose of adding a BN layer is to normalize the input data and meanwhile improve the training efficiency of the proposed SERR-U-Net. The equation of L2 regularization is as follows:

(3) $$\begin{array}{c} \underset{w}{\arg\min}L\left(w\right)=L_{\text{dice}}\left(w\right)+\lambda {\left\|w\right\|}_{2}^{2}. \end{array}$$

The L2 regularization is the value of *L*(*w*) plus the squared constraint of the L2 norm, where *L*_dice_(*w*) represents the loss function, and what this equation solves is the value of parameter *w* when the objective function *L*(*w*) gets the minimum value. L2 regularization can not only prevent overfitting, but also improve the generalization ability of the network, so as to segment the retinal vascular images more efficiently.

## 4. Experiments

### 4.1. Dataset

The experiments were conducted on two publicly available datasets DRIVE (https://http://drive.grand-challenge.org/DRIVE/) and STARE (http://cecas.clemson.edu/~ahoover/stare/probing). For the STARE dataset, it includes 20 JPEG retinal images. Ten of the images are of patients with no pathology (normals), and ten others contain pathology that obscures or confuses the blood vessel appearance in varying portions of the image (abnormals). The image resolution is 605 × 700, and each image corresponds to the manual annotated labels by two experts. For the DRIVE dataset, it includes 40 retinal images, 7 of which have symptoms of early diabetic retinopathy and 33 have no symptoms of diabetic retinopathy. Its image resolution is 565 × 584, and each image corresponds to the results manually annotated by two experts with masks. Considering that there are two manual segmentation results for the two public datasets, we select one result as the golden standard, and the other is used for qualitative comparison.

We manually divided the DRIVE and STARE datasets into training sets and test sets with the ratio of 1 : 1. The detailed division is shown in Table 2. For the DRIVE dataset, 20 images were used for training, and 20 images for test; meanwhile, four images were selected from the training set randomly for validation. For the STARE dataset, 10 images were selected for training, while 10 others for test; also, two images were selected from the training set randomly for validation.

Due to the limited amount of datasets in DRIVE and STARE, to reduce the influence of overfitting, in addition to the operations of L2 regularization and BN, the data augmentation is also implemented. By augmenting the DRIVE and STARE datasets, a set of 285,000 patches is obtained by extracting 9,500 patches for each training image.

### 4.2. Implementation

The experiments were implemented on a PC configured with Intel(R) Xeon(R) Silver 4110 CPU, GPU RTX 2080Ti, RAM 64G, Ubuntu 18.04, and the model was implemented using Python 3.7 and Keras 2.2.5 framework. In the training process, we use adaptive moment estimation (Adam) [28] as the optimizer and employ Tensorboard and Matplotlib for model visualization. The detailed training parameters are listed in Table 3.

### 4.3. Evaluation Metrics

To evaluate the performance of the proposed method, several metrics are used in this paper, including accuracy (ACC), sensitivity (SE), specificity (SP), and F1-score.

ACC is widely used for the task of binary classification, which is defined as the proportion of correct predictions (both true positives and true negatives) among the total number of cases examined. It is calculated as follows:

(4) $$\begin{array}{c} \text{ACC}=\frac{\text{TP}+\text{TN}}{\text{TP}+\text{TN}+\text{FP}+\text{FN}}, \end{array}$$

where TP, TN, FP, and FN represent true positive, true negative, false positive, and false negative, respectively.

SE is also called recall or true positive rate. It measures the proportion of actual positives that are correctly classified. It is calculated as follows:

(5) $$\begin{array}{c} \text{SE}\left(\frac{\text{recall}}{\text{true positive rate}}\right)=\frac{\text{TP}}{\text{TP}+\text{FN}}. \end{array}$$

SP is also referred as true negative rate, which measures the proportion of actual negatives that are correctly classified. It is calculated as follows:

(6) $$\begin{array}{c} \text{SP}\left(\text{true negative rate}\right)=\frac{\text{TN}}{\text{TN}+\text{FP}}. \end{array}$$

F1-score measures the balance between recall and precision, where precision calculates the proportion of true positives in the total predicted positive results. Precision is calculated as follows:

(7) $$\begin{array}{c} \text{Precision}=\frac{\text{TP}}{\text{TP}+\text{FP}}. \end{array}$$

The highest value of F1-score is 1.0, indicating perfect precision and recall, while the lowest value is 0, if either the precision or the recall is zero. F1-score is defined as follows:

(8) $$\begin{array}{c} \text{F}1=2*\frac{\text{precision}*\text{recall}}{\text{precision}+\text{recall}}=\frac{\text{TP}}{\text{TP}+1/2\left(\text{FP}+\text{FN}\right)}. \end{array}$$

Besides, since the receiver operating characteristic (ROC) curve is an important reference to measure the accuracy, it is also plotted with SP as the abscissa and SE as the ordinate. Moreover, the area under the curve (AUC) is utilized here, which is indicated by the area from the ROC curve to the two axes, and the closer the AUC is to 1, the better the performance.

In the training process, this paper uses the mean intersection over union (MIOU) for evaluation, but not for optimization. However, since it directly reflects the effect of the algorithm, thus it plays a guiding role in the following experiment. For a standard measure of semantic segmentation, it calculates the ratio of intersection over union as follows:

(9) $$\begin{array}{c} \text{MIOU}=\frac{1}{k+1}\overset{k}{\underset{i=0}{\sum }}\;\frac{\text{TP}}{\text{FN}+\text{FP}+\text{TP}}, \end{array}$$

in which *k* + 1 represents the number of categories.

### 4.4. Quantitative Analysis on Training Efficiency

Figure 6(a) shows the change of accuracy as the epoch increases during the training process. It can be seen that in the early stage, the network training curve converges quickly, and the learning efficiency of the model is higher. As training continues, the slope of the training curve decreases gradually, and the learning efficiency of the model slows down. When the number of training reaches about 13, the curve begins to be gradually parallel to the axis of abscissa, indicating that the learning efficiency of the network has reached saturation and appears slight fluctuation.

Regarding the selection of batch size, if it is too large, it would cause unstable and slow convergence and oscillating of loss value. On the contrary, it will lead to a large amount of calculation and high memory consumption. This experiment finally determines 25 for the batch size. Figures 6(b) and 6(b) show the change of loss and ACC as the batch increases, respectively. As the batch input reaches 16 k, the ACC peaks and the training loss drops to a minimum and stabilizes.

As the number of epoch increases continually (as shown in Figure 7(a)), the *loss* of training set gradually decreases after the 20th epoch; however, the *loss* of validation set increases. It is found a typical overfitting phenomenon, which is due to the excessive iterations of weight learning (overtraining) that fits the noise and the nonrepresentative features of the training image.

In this paper, we solve the overfitting problem by adding the BN layer and using L2 regularization. When only BN is added, the *loss* of validation set fluctuates as shown in Figure 7(b), while combined with L2 regularization, the loss of validation set decreases gradually as shown in Figure 7(c). Therefore, in the training, the BN layer enables a correlation of all the samples in an input batch; thus, the network would not generate a certain result from a specific training sample, but it will still produce *loss* fluctuation. Moreover, by adding L2 regularization on this basis can effectively avoid overfitting phenomenon.

### 4.5. Ablation Analysis

In this section, we conducted ablation experiments and analysis based on our SERR-U-Net code.

Table 4 shows the AUC and F1-score obtained by the network of different structures. For the U-Net, the final AUC is 0.9793, and the F1-score is 0.8360. For the recurrent+U-Net, the AUC of the network increases to 0.9799, and the F1-score increases to 0.8383. For the SE-ResNet+U-Net structure, the AUC of the network is 0.9834, and the F1-score is 0.8372. For the recurrent+ResNet+U-Net (R2-U-Net), the AUC and F1-score of the network increase to 0.9856 and 0.8474, respectively.

Compared to other structure, when the recurrent, SE, and ResNet structures are utilized together, the AUC of the network improves to the highest value of 0.9859, and the F1-score improves to the highest value of 0.8478, which indicates that the combination of the above structures enables a positive impact on the performance improvement of the other U-Net-based methods.

For an evaluation of the whole ablation, the ratio of AUC value F1-score was also calculated and shown in Figure 8, in which the abscissa and ordinate represent the AUC and the F1-score, respectively. The closer the bubble is to the upper right corner, the better the performance is. It can be seen that the bubble of our proposed method (purple) is located in the top right and thus proving a superior performance.

### 4.6. Test Results on DRIVE and STARE Datasets

This section conducts comparative experiments on the STARE and DRIVE retinal image datasets and compares the results of our proposed method with the contour manually annotated by one of the experts (expert 2^nd^ [9]).  Table 5 shows the comparative results with several metrics including ACC, AUC, SP, and SE.

As a result, the ACC of our proposed method is prior to the annotation of expert 2^nd^; however, the SP and SE of the proposed method on the DRIVE dataset are slightly lower than those manually annotated by expert 2^nd^. The main reason is that the proposed method is not as robust as that of expert 2^nd^ yet, especially at the intersection of small blood vessels.

Figures 9(b) and 9(c) illustrated some typical grayscale segmentation and binarization results on DRIVE dataset, while Figures 9(g) and 9(h) provided the typical grayscale segmentation and binarization results on STARE dataset.

By comparing the grayscale image, it can be seen that the proposed SERR-U-Net in this paper properly separated the vessel from its background and performed well both at the branch of the vessel and the endpoint of small blood vessel; thus, it is adaptable to the classification of multichannel images.

From Figures 9(d), 9(e), 9(h), and 9(i), we also found that both the proposed method could achieve vascular segmentation comparative to manual annotation. However, the manual labeling requires professional knowledge and patience. Moreover, the proposed method provided predication result with higher contrast than that annotated by manual depiction.

Table 6 provided the AUC results of the proposed method on the 20 DRIVE test images. It can be seen that the proposed model achieved a stable segmentation, with a minimal AUC value of 0.9618 and a maximal AUC value of 0.9874.  Table 7 showed the AUC results of the proposed method on 10 STARE images, with the minimal AUC value of 0.9826 and the maximal AUC value of 0.9899.

To demonstrate the changes of sensitivity and specificity of retinal vascular images with different thresholds, the ROC curve is depicted, which takes the false positive rate (FPR) as the abscissa and the true positive rate (TPR) as the ordinate.

Figure 10(a) shows the average ROC curve of the proposed method on the DRIVE dataset, and the average AUC reaches 0.9784.  Figure 10(b) shows the average ROC curve of the proposed method on the STARE dataset, and the average area under the curve (AUC) reaches 0.9859. The AUC values on both datasets are higher than that of U-Net, which proves a higher performance of the proposed method.

### 4.7. Qualitative Analysis on Intersection of Vessels and Small Vessels

In Figure 11, we select some intersections of vessels and the local area of small blood vessels to compare, in which the red box highlights the contrast of the segmentation effect of small blood vessels and vessel intersections.

By comparing the segmentation results of the original image (Figure 11(a)), the gold standard image (Figure 11(b)), the segmentation results of original U-Net (Figure 11(c)), and our proposed method (Figure 11(d)), we can see that the U-Net misclassifies some blood vessel area as the background at part of the small vessel and the branch of the vessel (indicated by blue arrow in Figure 11(c)), and the edge of the optic disc is incorrectly depicted as the blood vessels (indicated by red arrow in Figure 11(c)), which may cause negative impact on the clinical diagnosis.

The result is attributed to high-density downsampling of the proposed method, by which the feature information will not be excessively lost, so as to ensure that the segmentation of small blood vessels results in a higher accuracy, and the segmentation details of small blood vessels and intersections are retained to a greater extent, with a stable connectivity.

### 4.8. Quantitative Comparison with State-of-the-Art Methods

In order to further illustrate the performance of the proposed method in the retinal vessel segmentation, the method proposed in this paper is compared with some related state-of-the-art methods [29–34] with the aforementioned evaluation metrics.

In Table 8, based on DRIVE database, our proposed method obtained an ACC of 0.9552, SE of 0.7792, SP of 0.9813, and AUC of 0.9784. Compared with the unsupervised learning method [29–31], the proposed method performs better, mainly because the manually annotated labels are used to strengthen the training model, and thus, the reliability is higher. In addition, compared with the supervised learning method [32–34], although our SP is slightly lower than [32, 34], our other performances are superior.

In Table 9, based on the STARE database, our proposed method obtained an ACC of 0.9796, SE of 0.8220, SP of 0.9926, and AUC of 0.9859. Compared with the unsupervised learning method [29–31], our proposed method performs better, mainly due to the fact that the feature information is not excessively lost during the training process; thus, it is able to accurately identify the vascular features. Compared with the supervised learning method [32–34], the AUC value of the proposed method is slightly lower than that of [34]; however, our proposed method achieved superior performance on other performances.

The above results are mainly due to the ability of the proposed SERR-U-Net on deriving the context features, texture features, and other advanced features from the image. Specially, combined with SE, ResNet, and recurrent block, the network depth is increased by recurrent structure, and the attention mechanism is added to SE residual block to alleviate the gradient dispersion problem caused by the increase of network depth, and thus, the connectivity of small blood vessels and bifurcations is well retained.

## 5. Conclusions

Automatic segmentation of blood vessels from retinal images is a difficult problem in the field of medical image preprocessing, which is due to the lower contrast between the retinal vessels and the background, and uneven vessel width. This paper proposes a SERR-U-Net framework to improve the segmentation accuracy, which leverages the SE, ResNet, and recurrent technologies. The framework is supposed to derive more targeted feature information through SE and meanwhile employ residual structure to avoid the vanishing gradient problem caused by the increased network depth. The modified convolution layer enables high-density feature sampling to obtain vessel information of different sizes, which can properly represent the features of specific segmentation task.

The experimental results on DRIVE and STARE datasets show that the proposed method could achieve high accuracy that is comparable to manual annotation on retinal vascular segmentation. Specifically, it maintains a good performance in handling small blood vessels and blood vessel branches, which indicates a promising prospect in clinical assisted diagnosis. For the follow-up study, we would pay more attention on the segmentation method of retinal vascular with lesions and meanwhile reduce the training time.

## Figures and Tables

**Figure 1:** Flowchart of image preprocessing.

**Figure 2:** Individual channel representation of retinal images.

**Figure 3:** Random cropping of vessels: (a) original images and (b) annotated images.

**Figure 4:** The framework of the proposed SERR-U-Net.

**Figure 5:** Recurrent and residual module with attention mechanism.

**Figure 6:** Training visualization: (a) ACC with increasing epoch, (b) loss with increasing batch, and (c) ACC with increasing batch.

**Figure 7:** Overfitting analysis: (a) overfitting, (b) add BN layer, and (c) BN layer with L2 regularization.

**Figure 8:** Evaluation of ablation experiments on the 10 STARE images.

**Figure 9:** Segmentation results on DRIVE and STARE: (a, f) original retinal image; (b, g) grayscale conversion; (c, f) binarization; (d, i) our result; (e, j) expert 2^nd^.

**Figure 10:** ROC of different models for retinal vessel segmentation: (a) DRIVE and (b) STARE.

**Figure 11:** Comparative results of the proposed SEER-U-Net and U-Net: (a) original image, (b) golden standard, (c) result of U-Net (red arrow indicates the error at optic disc area, and blue arrow indicates the error at vessel branch area), and (d) result of our proposed method.

**Table 1:** Details of SERR-U-Net.

Block name	Layer (type)	Output size	Params
	Input (inputlayer)	(48, 48, 1)	0
Encoder block (1)	Conv2d_1 (Conv2D)	(48, 48, 16)	2320
	B_N(Batch Normalization)	(48, 48, 16)	64
SE_block_1 (SE-ResNet)			
Max_pooling2d (maxpooling2D)			
Encoder block (2)	Conv2d_2 (Conv2D)	(24, 24, 32)	9248
	B_N(Batch Normalization)	(24, 24, 32)	128
SE_block_2 (SE-ResNet)			
Max_pooling2d (maxpooling2D)			
Encoder block (3)	Conv2d_3 (Conv2D)	(12, 12, 64)	36928
	B_N(Batch Normalization)	(12, 12, 64)	256
SE_block_3 (SE-ResNet)			
Max_pooling2d (maxpooling2D)			
Encoder block (4)	Conv2d_4 (Conv2D)	(6, 6, 128)	147712
	B_N(Batch Normalization)	(6, 6, 128)	512
SE_block_4 (SE-ResNet)			
Encoder block (5)	Conv2d_5 (Conv2D)	(6, 6, 128)	147712
	B_N(Batch Normalization)	(6, 6, 128)	512
Up_sampling2d (upsampling2D)			
Decoder block (6)	Conv2d_6 (Conv2D)	(12, 12, 64)	36928
	B_N(Batch Normalization)	(12, 12, 64)	256
Up_sampling2d (upsampling2D)			
Decoder block (7)	Conv2d_7 (Conv2D)	(24, 24, 32)	9248
	B_N(Batch Normalization)	(24, 24, 32)	128
Up_sampling2d (upsampling2D)			
Decoder block (8)	Conv2d_8 (Conv2D)	(48, 48, 16)	2320
	B_N(Batch Normalization)	(48, 48, 16)	64
	Conv2d_9 (Conv2D)	(48, 48, 1)	0

**Table 2:** The division of datasets for training, validation, and test.

Database	Training	Validation	Test
DRIVE	20 images (190000 patches)	4 images (38000 patches)	20 images
STARE	10 images (95000 patches)	2 images (19000 patches)	10 images

**Table 3:** The detailed training parameters of implementation.

Parameters	Value
Learning rate	0.001
Learning step	5
Patch size	96 × 96
Downsampling ratio	500
Batch number	25
Epoch	20

**Table 4:** Comparing results of different ablation experiments on the 10 STARE images.

Methods	AUC	F1-score
U-Net	0.9793	0.8360
Recurrent+U-Net	0.9799	0.8383
SE-ResNet+U-Net	0.9834	0.8372
Recurrent+ResNet+U-Net (R2-U-Net)	0.9856	0.8474
Ours (SERR-U-Net)	0.9859	0.8478

**Table 5:** Comparative results between our proposed method and expert 2^nd^.

Database	Method	ACC	AUC	SP	SE
STARE	Ours	0.9796	0.9859	0.9926	0.8220
	Expert 2^nd^	0.9347	-	0.9382	0.8955
DRIVE	Ours	0.9552	0.9784	0.9813	0.7792
	Expert 2^nd^	0.9464	-	0.9717	0.7796

**Table 6:** AUC results of our proposed method on the 20 DRIVE images.

DRIVE	AUC	DRIVE	AUC	DRIVE	AUC	DRIVE	AUC
21_test.tif	0.9874	26_test.tif	0.9651	31_test.tif	0.977	36_test.tif	0.9862
22_test.tif	0.9824	27_test.tif	0.9796	32_test.tif	0.9618	37_test.tif	0.9831
23_test.tif	0.9624	28_test.tif	0.9758	33_test.tif	0.9772	38_test.tif	0.9842
24_test.tif	0.9756	29_test.tif	0.9789	34_test.tif	0.9824	39_test.tif	0.9838
25_test.tif	0.9768	30_test.tif	0.9772	35_test.tif	0.9780	40_test.tif	0.9841

**Table 7:** AUC results of our proposed method on the 10 STARE images.

STARE	AUC	STARE	AUC
im0081.ppm	0.9829	im0044.ppm	0.9870
im0291.ppm	0.9826	im0001.ppm	0.9881
im0005.ppm	0.9899	im0002.ppm	0.984
im0235.ppm	0.9866	im0255.ppm	0.9864
im0004.ppm	0.9832	im0236.ppm	0.9868

**Table 8:** Comparative results with state-of-the-art methods on DRIVE databases.

DRIVE	Methods	ACC	SE	SP	AUC
Unsupervised learning	Lam [29]	0.9472	\	\	0.9614
	You [30]	0.9434	0.7410	0.9751	\
	Azzopardi [31]	0.9442	0.7655	0.9704	0.9614
Supervised learning	Roychowdhury [32]	0.9520	0.7250	0.9830	0.9620
	Liskowsk [33]	0.9495	0.7763	0.9768	0.9720
	Qiaoliang [34]	0.9527	0.7569	0.9816	0.9738
	Ours	0.9552	0.7792	0.9813	0.9784

**Table 9:** Comparative results with state-of-the-art methods on STARE databases.

STARE	Methods	ACC	SE	SP	AUC
Unsupervised learning	Lam [29]	0.9567	\	\	0.9739
	You [30]	0.9497	0.7260	0.9756	\
	Azzopardi [31]	0.9563	0.7716	0.9701	0.9497
Supervised learning	Roychowdhury [32]	0.9510	0.7720	0.9730	0.9690
	Liskowsk [33]	0.9566	0.7867	0.9754	0.9785
	Qiaoliang [34]	0.9628	0.7726	0.9844	0.9879
	Ours	0.9796	0.8220	0.9926	0.9859

## Data Availability

The two datasets are publicly available as follows: DRIVE (https://drive.grand-challenge.org/DRIVE/) and STARE (http://cecas.clemson.edu/~ahoover/stare/probing).

## References

[1] Luo Z., Jia Y. (2020). The comparison of retinal vessel segmentation methods in retinal images. *Journal of Physics Conference Series*.

[2] Chaudhuri S., Chatterjee S., Katz N., Nelson M., Goldbaum M. (1989). Detection of blood vessels in retinal images using two-dimensional matched filters. *IEEE Transactions on Medical Imaging*.

[3] Yang Y., Huang S., Rao N. (2008). An automatic hybrid method for retinal blood vessel extraction. *International Journal of Applied Mathematics & Computer Science*.

[4] Zhao Y., Rada L., Chen K., Harding S. P., Zheng Y. (2015). Automated vessel segmentation using infinite perimeter active contour model with hybrid region information with application to retinal images. *IEEE Transactions on Medical Imaging*.

[5] Li Q., You J., Zhang D. (2012). Vessel segmentation and width estimation in retinal images using multiscale production of matched filter responses. *Expert Systems with Applications*.

[6] Staal J., Abramoff M. D., Niemeijer M., Viergever M. A., van Ginneken B. (2004). Ridge-based vessel segmentation in color images of the retina. *IEEE Transactions on Medical Imaging*.

[7] Soares J. V. B., Leandro J. J. G., Cesar R. M., Jelinek H. F., Cree M. J. (2006). Retinal vessel segmentation using the 2-D Gabor wavelet and supervised classification. *IEEE Transactions on Medical Imaging*.

[8] Ricci E., Perfetti R. (2007). Retinal blood vessel segmentation using line operators and support vector classification. *IEEE Transactions on Medical Imaging*.

[9] Fraz M. M., Remagnino P., Hoppe A. (2012). An ensemble classification-based approach applied to retinal blood vessel segmentation. *IEEE Transactions on Biomedical Engineering*.

[10] Fu H., Xu Y., Wong D. W. K., Liu J. Retinal vessel segmentation via deep learning network and fully-connected conditional random fields.

[11] Mo J., Zhang L. (2017). Multi-level deep supervised networks for retinal vessel segmentation. *International Journal of Computer Assisted Radiology and Surgery*.

[12] Jiang Y., Zhang H., Tan N., Chen L. (2019). Automatic retinal blood vessel segmentation based on fully convolutional neural networks. *Symmetry*.

[13] Dharmawan D. A., Li D., Ng B. P., Rahardja S. (2019). A new hybrid algorithm for retinal vessels segmentation on retinal images. *IEEE Access*.

[14] Brostow G. J., Fauqueur J., Cipolla R. (2009). Semantic object classes in video: A high-definition ground truth database. *Pattern Recognition Letters*.

[15] Lu D. (2020). Research on image recognition algorithm based on deep convolution neural network. *Academic Journal of Computing & Information Science*.

[16] Szegedy C., Liu W., Jia Y. Going deeper with convolutions.

[17] He K., Zhang X., Ren S., Sun J. Identity mappings in deep residual networks.

[18] Ronneberger O., Fischer P., Brox T. U-Net: convolutional networks for biomedical image segmentation.

[19] Milletari F., Navab N., Ahmadi S. A. V-Net: fully convolutional neural networks for volumetric medical image segmentation.

[20] Lai S., Xu L., Liu K., Zhao J. Recurrent convolutional neural networks for text classification.

[21] Szegedy C., Ioffe S., Vanhoucke V., Alemi A. A. Inception-v4, inception-resnet and the impact of residual connections on learning.

[22] Lian S., Li L., Lian G., Xiao X., Luo Z., Li S. (2021). A global and local enhanced residual U-Net for accurate retinal vessel segmentation. *IEEE/ACM Transactions on Computational Biology and Bioinformatics*.

[23] Hu J., Shen L., Sun G. Squeeze-and-excitation networks.

[24] Guo C., Szemenyei M., Yi Y., Zhou W., Bian H. Residual spatial attention network for retinal vessel segmentation.

[25] Wang X., Yu K., Wu S. Esrgan: enhanced super-resolution generative adversarial networks.

[26] Alom M. Z., Hasan M., Yakopcic C., Taha T. M., Asari V. K. (2018). Recurrent residual convolutional neural network based on U-Net (r2U-Net) for medical image segmentation. https://arxiv.org/abs/1802.06955.

[27] Soomro T. A., Afifi A. J., Gao J., Hellwich O., Paul M., Zheng L. Strided U-Net model: retinal vessels segmentation using dice loss.

[28] Newey W. K. (1988). Adaptive estimation of regression models via moment restrictions. *Journal of Econometrics*.

[29] Lam B. S. Y., Yongsheng Gao, Liew W. C. (2010). General retinal vessel segmentation using regularization-based multiconcavity modeling. *IEEE Transactions on Medical Imaging*.

[30] You X., Peng Q., Yuan Y., Cheung Y. M., Lei J. (2011). Segmentation of retinal blood vessels using the radial projection and semi- supervised approach. *Pattern Recognition*.

[31] Azzopardi G., Strisciuglio N., Vento M., Petkov N. (2015). Trainable COSFIRE filters for vessel delineation with application to retinal images. *Medical Image Analysis*.

[32] Roychowdhury S., Koozekanani D., Parhi K. (2014). Blood vessel segmentation of fundus images by major vessel extraction and subimage classification. *IEEE Journal of Biomedical and Health Informatics*.

[33] Liskowski P., Krawiec K. (2016). Segmenting retinal blood vessels with deep neural networks. *IEEE Transactions on Medical Imaging*.

[34] Li Q., Feng B., Xie L. P., Liang P., Zhang H., Wang T. (2016). A cross-modality learning approach for vessel segmentation in retinal images. *IEEE Transactions on Medical Imaging*.

